The article "Long Jump Action Recognition Based on Deep Convolutional Neural Network" was retracted in 2023. Reasons: signs of a paper mill; suspected computer-generated content; unreliable results or conclusions; lack of ethics approval or compliance.

# Long Jump Action Recognition Based on Deep Convolutional Neural Network

**DOI:** 10.1155/2022/3832118

**Published:** 2022-05-29

**Authors:** Zhiteng Wang

**Affiliations:** Fujian Normal University, Fuzhou 350108, Fujian, China

## Abstract

Long jump is a test item of national student physical health monitoring, which can reflect the quality of students' lower limb strength. Long jump is a highly technical activity, which includes four basic movements: running aid, jumping, vacating, and landing. Many students have problems with the technical aspects, resulting in test scores that do not objectively reflect the true physical condition of the students, which affects the accuracy of the test results. From the perspective of rapid diagnostic feedback of students' long jump movements, we design and develop a long jump movement recognition method based on deep convolutional neural network. In this paper, we firstly summarize the traditional visual action recognition algorithm, then apply 3D convolution to extract the spatiotemporal features of long jump action from three directions of the video block, and fuse the spatiotemporal features of the three directions in different ways to achieve feature complementation; finally, using the multimodality of long jump action data, we use 3D convolutional neural network to train the RGB images and then train the depth. This joint training method can accelerate the convergence speed and improve the accuracy of the network on both depth and edge images. The experiments compared the recognition effects of the tandem fusion of features, the maximum fusion, and the multiplicative fusion in the scoring layer, and the highest accuracy of 82.3% was achieved by the tandem fusion of features with the fusion of three modalities.

## 1. Introduction

Students' physical health is a hot issue of national and social concern at present. The testing and data reporting of students' physical fitness has become a regular task of all universities in China every year. In the test of students' physical health, long jump, as a test item reflecting students' lower limb strength, occupies 10% weight in the whole test and is an important item in the physical health test. In the current track and field general education course, long jump is one of the key items for students to learn, mainly based on the teaching of jerk long jump, supplemented by the explanation and introduction of walking long jump teaching [1]. However, the teaching of long jump technique is often not given enough attention, so how to make students control the reasonable and complete long jump technique within the limited teaching hours is a practical problem faced by long jump teaching for a long time.

With the in-depth research on long jump teaching, there are more and more studies on the application of teaching methods in long jump classrooms. Hou proposed to integrate PBL teaching method into the classroom of long jump teaching. This teaching method is to advocate the student as the main body and teacher as the leader and to ask problems to guide students to solve problems. By asking questions and then solving problems, students can improve their learning initiative and learn how to learn. After experimental verification, the application of PBL method to long jump teaching can improve students' skills in problem identification, problem analysis, and problem solving, as well as improving students' ability to learn skills and theories and their ability to innovate. Applying the structure-directed teaching theory to the long jump lecture, Lu mentioned that the structure-directed teaching model is an effective supplement to the traditional teaching methods, so it also points out an effective but not the only method for the long jump lecture classroom. The introduction of the structural-directed teaching model into the classroom lectures is done using its orientation to the psychological structure of the students and combining it with contemporary research findings in various aspects of information technology, theory, and methodology and a new way of teaching long jump combining experiment and theory [2]. The results show that this type of teaching model is more suitable for teaching long jump, and the learning of movement skills under this teaching model has the characteristics of long term and stability. King proposed a classification method for long jump technique, as shown in Figure 1.

The procedure of teaching long jump technique was developed by combining procedural teaching method and spatiotemporal cognition. This procedure is based on an in-depth study of the connection between theoretical basis, teaching objectives, teaching principles, and teaching evaluation and the analysis of relevant conclusions. Then, through a 20-hour teaching experiment, a comparative study was conducted on the attainment and technical assessment scores of students in the experimental and control groups, as well as on the problems of observation, analysis, problem solving, and cognitive ability. Good effects were found in improving students' motivation to learn as well as their thinking skills. Guo proposed to introduce the task-driven teaching method into the general track and field course of the physical education faculty and analyzed the data results before and after the experiment by conducting an experimental study on track and field teaching, which is guided by the theory of track and field teaching. Its teacher-led principle, student-main principle, task-main principle, and competence theme principle are reflected in all aspects of the teaching design activities of the general track and field course and become the basic guidelines for guiding teaching activities [3]. The experimental study found that although there was no difference in physical form and physical quality, the experimental group was more prominent in terms of learning motivation, self-confidence, sense of accomplishment, and the performance of long jump skill improvement. It shows that the task-driven teaching method can significantly improve the teaching effect when used for teaching track and field.

In today's teaching, the “practice method” is the main method, supplemented by lecture, demonstration, and error prevention and correction methods, which is too boring and monotonous and lacks the grasp of the actual teaching situation and effective guidance. In the technical action diagnosis of physical education and sports training, the recording and analysis of human kinematic parameters based on video analysis or 3D motion capture technology can quantify the kinematic characteristics of technical actions and then discover the action problems and provide scientific suggestions for action improvement [4]. However, video analysis and 3D motion capture methods are complicated, and the data testing and analysis period is long, which cannot realize the technical diagnosis task for a larger number of students in a short period of time, so it is difficult to be applied in a large scale in students' long jump technical movements. Machine vision-based motion recognition methods provide a solution to this problem. The most used information in vision-based human-computer interaction is face and movement, and body movements are widely used in various intelligent interactive products by virtue of their natural, rich, and comfortable performance characteristics. Motion recognition is dynamic in nature and has uncertainty in space and time, which makes it more difficult to recognize. The research on vision-based action recognition is divided into two categories: one is the traditional action recognition method, which includes four stages of action segmentation, action tracking, action feature extraction, and action classification, each of which requires very strict algorithms; the other is the action recognition based on convolutional neural network [5]. After years of research, many technologies of action recognition have been practically applied. In 1996, IBM launched a game device based on acceleration sensor; in 2006, Japan's Nintendo added sensors to the game controller to capture body movement, enhancing the game experience; then the Israeli 3D sensor company Primesense developed a 3-dimensional structured light principle of the camera Microsoft used to develop the earliest Kinect, so that body interaction has become a research hot spot; in 2012, the company launched a new generation of 3D sensors Capri, as the smallest sensor at the time, with low price and low power consumption, becoming the first 3D sensor that can be widely used in smart phones and tablets. Israeli company eyeSight in the 2016 World Congress of Communication released a smart home system called sing cue IoT shine; users can control the volume of audio, lighting, and multimedia playback in the home through hand body movements. LeapFMotion developed a body-sensing controller, which can be connected to a PC, allowing users to browse the web, play PPT, and access information through finger movements.

Based on some classic research theories, the main contributions of this paper are as follows: (1) A 3D convolutional neural network with multimodal joint training and a 3D convolutional neural network with multidirectional feature fusion is proposed for long jump action recognition, providing students with rapid diagnosis of technical movements in the long jump. (2) The proposed three-dimensional convolutional neural network is used for long jump action recognition, which can quickly diagnose students' long jump technical actions. (3) It provides targeted advice for action improvement.

## 2. Related Works

### 2.1. Current Status of Long Jump Technology Research

In today's world, the difference in performance between athletes is very close. In domestic athletics competitions, the difference of a few centimeters often determines the winner of the whole long jump competition. Many athletes with good strength lose the long jump championship just because of the bad accuracy of long jump assist. Liang talked about the analysis of the factors influencing the accuracy of long jump assisted jump in “Discussion on the accuracy of long jump assisted jump”; she believed that the factors influencing the accuracy of long jump assisted jump are divided into four aspects, namely, the way of start, acceleration, rhythm, and psychological factors. These four factors should be taken into consideration and the training should be carried out according to the individual characteristics of the athletes. Another important point in the study of the factors influencing the accuracy of running aid is that many traditional sports coaches ignore the importance of teaching running aid in physical education and do not establish a reasonable structure system of running aid in students' hearts. However, the traditional long jump running aid practice only pays attention to the jumping technique and aerial movements but neglects the practice of athletes' running aid rate. Based on the factors that affect the accuracy of long jump assist, Zhang also pointed out to the environment in her article [6]. She believes that the environment is also an aspect that has a great impact on the accuracy of the long jump. James pointed out that athletes should correct their body posture, stride frequency, and stride length in the last 3-2 steps; it is beneficial to coordinate stride length through visual perception in the last few steps to improve the pedaling technique. Brigitte's findings also suggest that the athlete's accurate visual control of the limbs to achieve perfect coordination also plays an important role in the final accuracy on the board. In his article, Jing Summit mentions the appropriate rhythm of the assist, which he believes to be an acceleration of the assist, reaching the highest rate of the assist in the last few steps and the acceleration of the rate of the assist in the last few steps lies in the acceleration of the stride frequency. However, whether the assisted running reaches its highest speed which is the perfect assisted running speed, it can get a beautiful sports performance. Based on this problem, the answer is given in Xu's “Exploration of long jump assisted running rhythm pattern”; he favors that the assisted running speed of long jump determines the performance of long jump to a great extent, which has also been confirmed. By reviewing the information, we found that many excellent long jumpers did not reach their top speed when they set their best performance [7]. In addition to obtaining a top horizontal speed, the long jump assist has to prepare for stepping onto the springboard. So Xu pointed out that the long jump assisted running speed is not their highest speed, but in the process of assisted running they constantly find a suitable assisted running rate, with a suitable, scientific assisted running speed for long jump sports to get good results. The flowchart of vision-based action recognition is shown in Figure 2.

Long jump speed utilization refers to the long jumper's use of his own rate when performing long jump running aid. Many people have conducted research on the use of long jump assist and the effect on the assist rate. According to our scholars for more than ten years to monitor the utilization rate of the assisted running speed it can be seen that most of our long jumpers jump utilization rate reached 97%-98%, while most foreign high-level long jumpers jump utilization rate is only 93%–95%, This proves that our long jumpers are constantly improving their jumping utilization rate in order to pursue faster running speed and better long jump achievement. However, the final result is also unsatisfactory; however, through the statistics it can be concluded that our athletes' assisted running utilization rate reaches more than 98%, while foreign players are only about 94%, but why is our performance worse than foreign players? This has formed a huge reaction in the long jump community, overturning the basic theory of our researchers on the pursuit of speed and speed utilization rate as the core. It is not the case that a large speed utilization rate of assisted running will be conducive to obtaining the desired results. In 2004, Wang published an article on “Exploring the utilization rate of running speed in long jump” in the Capital Sports Journal and proposed the concept of the possibility of adopting a lower utilization rate of running speed [8]. People are now questioning the utilization rate of excessive running speed, and this issue still needs further research and discovery. The continuous development of science and technology has always been in the continuous breaking through the old ideas and theories, without the exploration of the old ideas there will be no new understanding, the birth of a new theory.

The jumping technique is the focus of the whole long jump, and it is also a very important step in determining the long jump performance. The initial speed and angle of takeoff directly determine the distance of long jump, and the instantaneous jump determines the horizontal and vertical rates. While the horizontal speed is determined by the difference between the assisted speed and the horizontal speed lost during the jump, the vertical speed is determined by the instantaneous speed during the jump. The jumping technique needs to be done with fast pedaling and positive cushioning as well as a strong swinging action of the swinging leg to be able to complete the jump quickly. In his article, Jia discusses jumping technique as the main indicator of long jump technique. He advocates that the loss of horizontal speed will lead to poor stability of the technical movement in the jumping phase, and the time of pedal extension is too short, which eventually affects the jumping result. Shepherd suggests in his article “Long Jump Technique” that the teaching of long jump technique should be taught and practiced separately for each part of the technique [9]. When teachers teach long jump, special emphasis should be placed on teaching the connection between running and jumping.

Research at home and abroad proves that, without the influence of external forces, the trajectory of human center of gravity should not change when long jump is in the air, and the series of body movement techniques of long jumpers after the air is actually to maintain the balance of the body and make sufficient preparation for a better landing. Chen research on the technology of modern men's long jump and its training characteristics shows that the landing technology has little effect on the performance of high jump, and the correct landing technology can effectively protect the body from injury, and when landing, the belly should be well lifted and legs collected, and the timing of bending knee buffer should be mastered. To sum up, in the study of long jump technique, in order to improve students' motivation and enhance the teaching efficiency of the classroom, many physical education teachers have proposed a variety of teaching methods that can be reasonably incorporated into the long jump classroom [10], for example, the PBL method, the Structure-Orientation method, the Goal-Setting method, the Procedural method, the Nimble method, and the Mutual Learning method. With these methods Wei later laid the theoretical and practical foundation for teaching; however, there is no in-depth research analysis, systematic design, and research application for beginners learning long jump technique.

### 2.2. Current Status of Action Recognition Research

Currently, deep learning-based action recognition networks mainly include 2D CNN, 3D CNN, and spatiotemporal decomposition networks according to the characteristics of the backbone network. The action recognition method based on 2D CNN has gone through two main research phases: the first phase, based on dual-stream networks, and the second phase, based on 2D CNN, by effectively building temporal feature extraction modules to capture temporal contextual information so as to avoid the input of optical streams. Phase I: In response to the problem that single-stream 2D CNNs cannot model temporal information, Simonyan proposes a dual-stream network [11]. For training, the spatial flow network and the temporal flow network are trained separately. For testing, the softmax scores of the two streams are aggregated by averaging all sampled video frames to obtain video-level prediction results. The drawbacks of the traditional dual-stream network are as follows: (1) since optical streams only represent motion information between adjacent frames, the dual-stream network has very limited access to temporal context, which is not conducive to modeling some movements with large time spans; (2) compared with the traditional dual-stream network, LSTM can more effectively represent the dependencies of video frames on time sequences, thus enabling the modeling of long-time sequences. However, its modeling of the underlying temporal information between video frames is inadequate, resulting in the loss of temporal information, and the introduction of LSTM leads to a large amount of computational overhead, which is not conducive to the optimization of the network at a later stage. Therefore, Wang proposed a time-domain segmentation network. TSN introduces a sparse sampling strategy based on a dual-stream network by first segmenting the input video into several segments and then randomly sampling one frame from each segment, and each frame is independently extracted by CNN for spatiotemporal features [12]. The outputs of each segment are combined using segment consensus functions to obtain consensus between segments regarding category assumptions. Finally, the category scores of spatial and temporal streams are fused to obtain video-level predictions. The sparse sampling strategy of TSN ensures that the input frames cover each time segment in the video, and this video-level supervised approach gives the network the ability to extract global spatiotemporal features, effectively solving the problem of traditional dual-stream networks lacking the ability to model long-time structures. However, not all randomly sampled segments contain information related to action recognition, so Lan proposes a self-learning weighted fusion method based on TSN, where the weights of each segment are obtained by the network autonomously learning, effectively solving the problem of unreasonable weight assignment in TSN. Phase 2: Zhu proposes an implicit dual flow network. It can implicitly capture the motion information between adjacent frames without precomputing optical flow, which saves storage space and speeds up the operation of the algorithm. Sun proposes an optical flow-guided feature, which extracts the optical flow-guided features at different levels by calculating the spatial gradients of the horizontal and vertical directions of the feature maps and the temporal gradients between different feature maps, so that the CNN can directly capture the temporal information between different temporal information between frames directly. In addition, Lee proposed a motion feature network for modeling the spatiotemporal information between consecutive frames. MFNet consists of appearance blocks encoding spatial information and motion blocks encoding temporal information. Among them, the motion block takes the feature maps of adjacent times as input and uses motion filters instead of shift operations between spatial feature maps for modeling the computational process of optical flow. Another idea is to process the information on the time channel efficiently to capture the temporal cues between feature maps. For example, Lin proposes a time-shift module for processing temporal information. It blends temporal information on adjacent feature maps by channel shift operations on the temporal domain, and the temporal perceptual field is correspondingly expanded by a factor of two for modeling a one-dimensional convolution with a temporal kernel size of 3 for the purpose of modeling temporal features [13]. The 2D convolutional interchannel fusion capability is also utilized for the original temporal fusion, making the 2D CNN capable of capturing temporal cues without incurring additional computational cost. The process of action segmentation based on contour information is shown in Figure 3.

The architecture obtains grayscale, gradient, and optical channel information from adjacent frames in the video, then convolves and downsamples each channel separately, and finally combines the information of all channels to obtain the final feature representation. Inspired by the excellent performance of residual networks in the field of image classification, Tran extended the C3D architecture to deep residual networks and proposed the Res3D network. By varying the number of filters in each convolutional layer to keep the parameters of the network architecture consistent, the effects of the sampling frequency of the input frames, the spatial resolution, and the type of convolution on the model performance are explored. Meanwhile, the number of parameters and computational complexity of Res3D are 1/2 of those of C3D, and the top-1 and top-5 on the Sport-1M dataset are improved by 4.5 and 2.6 percentage points, respectively. T-C3D introduces the video-level supervision method of TSN, while ensuring that the 3D CNNs of each segment share weights, which is beneficial to obtain global spatiotemporal features without generating additional parameters. In addition, the use of an attention pool as a segment consensus function enables the network to efficiently distinguish the importance of each input segment, which greatly improves the performance of the model [14]. By deploying an additional jump connection between adjacent residual blocks, Wang not only fully integrates the shallow and deep spatiotemporal features, but also effectively mitigates the gradient disappearance and overfitting that 3D CNNs tend to produce as the network deepens. Qian explores the impact of five convex strategies on residual learning by customizing the jump connection coefficients of the residual network. Carreira extends the Inception network using 3D convolution and pooling operations to propose I3D, which uses a larger spatiotemporal resolution for the input of the I3D network, and proposes a new method of initializing 3D CNNs. The weights of the 2D filters initialized by ImageNet are extended along the temporal dimension while dividing by the number of extensions to ensure the same dimensional response of the filters. Meanwhile, pretraining on the Kinetics dataset and fine-tuning on the UCF101 and HMDB51 datasets yielded 98.0% and 80.7% accuracy, respectively. However, I3D is extremely demanding in terms of hardware configuration because it uses a large number of input frames and optical flow images for training and testing. Unlike the above networks that learn spatiotemporal features in short clips (16 frames), Varol proposes the LTC network for the problem that it is difficult for local 3D convolution to model spatiotemporal features in inputs with long action durations. The main idea is to maintain the parameter balance by decreasing the spatial resolution of the input frames to increase their temporal resolution and verify the effect of long input time on the performance of the action recognition model. The 3D CNN uses 3D convolution to capture spatiotemporal information simultaneously and is able to process multiple input frames at a time, so the algorithm runs faster. However, 3D convolution introduces a large number of parameters, which results in high computational cost and memory overhead [15]. Most of the current 3D CNN-based methods combine the idea of dual-stream networks, using optical stream images as input to enhance the performance of the model.

Spatiotemporal decomposition networks mainly include spatiotemporal decomposition convolution that decouples spatiotemporal filters and channel separation convolution that separates spatiotemporal feature channels. Based on this, Qiu proposes a pseudo-3D residual network, which further reduces the number of parameters by introducing bottleneck architectures at both ends of the 1 × 3 × 3 and 3 × 1 × 1 convolutions for reducing and recovering the dimensionality of the input feature maps. Three pseudo-3D residual units were constructed using three jump connection patterns, cascade, serial, and cascade and serial, for representing the direct or indirect influence existing between spatial and temporal filters. By introducing the bottleneck block architecture and spatiotemporal decomposition convolution, P3D can be embedded into ResNet-152, which greatly extends the depth of the network. Xie, on the other hand, has transformed the I3D network by spatiotemporal decomposition convolution and proposed the S3D network. The network of S3D by spatiotemporal decoupling has fewer parameters and less computational complexity compared to the I3D network. Meanwhile, the top-1 accuracy is improved by 1.1 percentage points and 1.5 percentage points on the Kinetics dataset and something dataset, respectively, further verifying that the spatiotemporal decoupled convolution is more favorable to allocate parameter space and has better spatiotemporal modeling ability [16]. In addition, Li proposed a collaborative spatiotemporal module to encode spatiotemporal features collaboratively by applying weight sharing constraints to the learnable parameters. Unlike the above methods that reduce network parameters by decoupling spatiotemporal filters, the use of channel grouped convolution can effectively reduce the number of spatiotemporal interactions, thus reducing the temporal complexity of the network. Luo proposes a grouped spatiotemporal aggregation approach. Gst decomposes feature channels into spatial and temporal groups in parallel, with the spatial group using 2D convolution for capturing appearance cues and the temporal group using 3D convolution for capturing temporal cues. With asymmetric channel decomposition, GST can qualitatively analyze the importance of temporal and spatial features at different stages by visualizing the scale factor of each channel in the regularization layer, so as to understand how spatial and temporal cues are encoded from the underlying features to the higher-level features. Considering the complementarities of spatiotemporal and motion features, Jiang proposes a spatiotemporal and motion coding. The STM uses two-dimensional spatial convolution and one-dimensional temporal convolution to separate modeled spatiotemporal features by reorganizing the input channels; the channeled motion module performs feature differencing of adjacent feature maps in the temporal dimension for extracting feature-level motion patterns between adjacent frames and greatly reduces the memory consumption.

## 3. Algorithm Design

### 3.1. Model Structure

After decades of development, the vision-based action recognition system has been very mature, with the main recognition process in the system. In the traditional method, the continuous image sequence is firstly collected by the video acquisition terminal and sent to the computer, then the action in the image sequence is extracted from the complex background by the action segmentation algorithm, then the motion information of the action is obtained by the target tracking algorithm, including the spatial action change and the temporal action trajectory, then the spatiotemporal features of the whole image sequence are extracted by the manually designed feature extraction algorithm, and finally, various classifier algorithms are used to classify the features.

#### 3.1.1. Action Segmentation

A good action segmentation algorithm is crucial, because the subsequent processing will depend on the results of action segmentation. At present, researchers have conducted in-depth research on action segmentation algorithms based on skin color, motion information, contour, and other information, which are applied to different environmental scenes.

The skin color-based action segmentation is the most useful algorithm when the contrast between background color and skin color is large. The YCbCr space is the most used color space for skin color detection. Compared with RGB color space, YCbCr space separates luminance and color, which can restrict the area of skin color distribution, and the effect of skin color clustering is obvious, which can meet the requirements of different skin color segmentation [17]. At present, in YCbCr space, mixed Gaussian model, and probability model are the most commonly used skin color segmentation models. The most widely used one is the skin color ellipse model proposed by Rein et al. which was first applied to face segmentation, and then Fang used the skin color ellipse model for static action segmentation. However, the main drawback of the skin color-based action segmentation algorithm is that it is less effective when there are near-skinned targets in the background or when the image contains other skin-colored organs such as faces. Therefore, in order to improve the accuracy of segmentation, it is generally used in combination with motion information-based and contour-based segmentation algorithms.

Motion information-based motion segmentation is mainly used in video to segment the continuously changing motion. In the video, the action is the main motion target, and the background is usually stationary, so some motion target detection algorithms can locate the action and segment the action from the background. In addition, researchers have also proposed some background modeling algorithms, such as Kalman filtering method, hybrid Gaussian modeling method, and statistical averaging method. The optical flow method maps the motion of the target in 3D space to the change of pixels on a flat image and obtains the motion information of the target by calculating the motion speed of pixels in the image, which can accurately obtain the motion information of each pixel compared with other methods, but the disadvantage is that the algorithm is more complicated. The motion segmentation algorithm based on motion information also has obvious shortcomings, when there are motion targets other than motion in the video; the effect of motion segmentation is often unsatisfactory.

As the unique feature of the limb, the action segmentation based on contour information can avoid the impact of different races and skin tones compared with other segmentation methods and also have certain robustness to lighting changes. Currently, the widely used methods are edge detection and contour template matching. The edge detection method obtains the edge of the action by the edge detection operator, which is mainly suitable for images with simple background. When the background is more complex, the background edges will strongly interfere with the action edges. The template matching method is to locate the action by traversing the predefined action template on the image to be detected and calculating the match with all the targets on the image [18]. However, due to the variety of actions, there is no fixed template for the action, and it is computationally expensive to traverse the whole image, so scholars gradually give up using template matching method for action segmentation. There are also action segmentation algorithms based on active contour model, visual saliency, and full convolutional neural network, which have their own advantages and disadvantages and are generally a combination of multiple segmentation algorithms to achieve complementary advantages.

#### 3.1.2. Motion Tracking

Motion tracking can be used either as a step in motion recognition or as a standalone application in human-computer interaction, such as controlling the movement of the mouse by tracking the motion. Motion tracking first obtains the action to be tracked in the first frame of the video through the action segmentation algorithm and then uses the action tracking algorithm to continuously locate the action in subsequent frames, so the action tracking functionally replaces the action segmentation in subsequent video frames. The action tracking effect can also be achieved by doing action segmentation on each frame of the video, but the action segmentation algorithm is computationally intensive and cannot achieve real-time requirements. Currently, researchers have developed two target tracking algorithms based on modeling methods for tracking targets: generative tracking and discriminative tracking.

The generative model tracking algorithm first extracts features such as Hu moment features and color features from the target, then traverses the whole image, and measures the similarity between the features extracted from an area of the image and the features of the target to be tracked. This operation is performed continuously for each frame in the video to achieve the target tracking. The classical generative model tracking algorithms are mean shift, Kalman filter, and particle method, etc. Mean shift algorithm is the simplest tracking algorithm, and its tracking process is shown in Figure 4. The disadvantage of the mean shift algorithm is that it is easy to lose the target when the target outline is similar to the background; the tracking effect becomes worse when there is a near-skinned object in the background.

The discriminative model tracking classifies the pixels in the foreground and background of each frame of the video. When tracking the target, the pixels in the current frame are used as positive samples and the negative samples are used as background regions to train the classifier, which is then used to find similar regions as target regions in the next frame and then repeated in subsequent frames to complete the tracking of the target. Currently the more popular discriminative tracking algorithms are Struck algorithm and TLD algorithm. Firstly, the static action detection is performed by HAAR cascade classifier, then the action is tracked and the action trajectory is extracted by the improved TLD algorithm, and finally the dynamic action recognition is completed by the improved DTW algorithm. Zhang introduced Kalman filter and hidden Markov model in the TLD algorithm to solve the occlusion problem of action tracking and improve the processing speed.

#### 3.1.3. Action Feature Extraction

In action recognition, how to efficiently extract the target features to remove redundant data is crucial to the final recognition result, and action recognition is no exception. Features are not precisely defined in the image field but are generally understood to represent a segment of the image coding, and the features extracted from different categories of images have high variability and reliability. In addition, feature extraction allows images to change from high-dimensional data to low-dimensional data, removing redundant data, thus speeding up recognition and improving recognition accuracy. Static action feature extraction only needs to focus on the spatial changes on the limbs, while dynamic action feature extraction extracts spatial plus temporal features from the image sequence, which must be combined with the upper and lower adjacent frames, making feature extraction more difficult. Currently, in video classification including action recognition, the range of features can be divided into global features and local features.

Global features are extracted by first locating or segmenting the object from the image before extracting features, and then some kind of feature extraction is performed to form global features. The global feature is very effective; it contains all the information of the object, including the topology between the various parts of the object such as the relative position of multiple actions [19]. Bhanu was the first to use contour features to describe human actions and introduced the motion energy map, and in order to achieve a better feature description, the motion history map was proposed based on Bhanu's improved algorithm.

Local feature extraction is a bottom-up feature extraction of the local part of the target. The first step is to extract some spatiotemporal key points in the video, also called interest points, and then further compute the regions where these key points are located to obtain image blocks, and finally combine these image blocks to describe a specific action. The advantage of local features is that they do not depend on target segmentation, localization, and tracking and are insensitive to noise and occlusion. However, local features require a large number of stable spatiotemporal interest points as support and are computationally intensive in the preprocessing stage. French researcher NavneetFDalai proposed the histogram of gradient direction algorithm. HOG is to count the gradient information of pixels in an image. Its main steps are as follows: firstly, multiple pixels in the image are formed into a cell, and the gradient information of each cell is calculated, then multiple cells are formed into a block, and the gradient histogram of a block is generated; finally, the gradient histogram of all blocks is combined and contrast normalized to get the final HOG features.

#### 3.1.4. Convolution-Based Action Recognition

Convolutional neural network (CNN) is a nonlinear mathematical model designed by human to imitate the visual properties of animals and neural transmission in the brain, which can map raw data such as images and sounds through multiple layers of nonlinear kernel functions to generate high-level feature representations that are more discriminative than the original data. In 1989, LeCun proposed the first LeNet model similar to the modern network structure for handwriting classification and introduced the term “convolution” in his paper. Since then, the theoretical research and application of convolutional neural networks have been stagnant due to the lack of hardware computing power and data samples. It was not until 2012 that AlexNet won the ImageNet challenge that convolutional neural networks became a hot topic for academic research again [20]. With the increase of GPU computing power, the network structure has developed in a deeper direction from 8-layer AlexNet to 16-layer VGGNet to 152-layer ResNet. These classical network models are similar in that they are composed of convolutional layers, nonlinear mapping layers, and pooling layers, which are alternately connected and finally classified by a fully connected layer.

The main function of the convolutional layer in a convolutional neural network is to extract features by convolving the feature map with the convolutional kernel of the current layer and then send the generated new feature map to the next convolutional layer. In order to reduce the overfitting of the network and improve the generalization ability of the neural network, the convolutional layer is locally connected; a neuron does not need to connect to all the feature points in the feature map, but only to the local area adjacent to it. The nonlinear mapping layer consists of various activation functions and is the core layer of the deep convolutional neural network. Obviously, the role of the nonlinear mapping layer is to provide the convolutional neural network with the ability of nonlinear variation and to enhance the feature expression of the network by cascading multiple layers of nonlinear mapping layers. Without the nonlinear mapping layer, no matter how deep the convolutional neural network is, the final extracted features are linear mapping of the original data, which cannot solve the problem of classifying nonlinearly separable data [21]. The pooling layer, also known as the downsampling layer, generally follows the nonlinear mapping layer, and its main function is to reduce the size of the feature map, thus reducing the number of model parameters, in addition to reducing the risk of overfitting and improving the generalization ability of the network.

After the multiple convolutional layers are used for nonlinear mapping of the input image, the extracted features are already very abstract. At this time, traditional machine learning methods such as SVM, decision tree, and random forest can be chosen for classification, while in the convolutional neural network, the classification is performed by fully connected layers. The standard connection of fully connected layers is shown in Figure 5, where the neurons in the front and back layers are fully connected and the features to be classified are mapped to the sample labels by a linear transformation called weighted summation. The number of neurons in the fully connected layer is crucial because of the fully connected nature of the fully connected layer, which is the source of more than 90% of the training parameters of the convolutional neural network.

In general, the number of neurons in the fully connected layer is set to be large, and then the dropout technique is used to reduce the overfitting of the network model in Figure 6. The number of parameters is greatly reduced by not involving the neuron in the forward computation and backward propagation of the network. At the same time, the role of the original fixed-connected design elements in updating the weights is reduced, and the network learns more robust features.

After the introduction of AlexNet network, deep convolutional neural networks have been widely used in various image tasks such as object recognition, target segmentation and detection, and image saliency detection. During this period, some classical network structures such as VGG, GoogLenet, and ResNet have also emerged. In view of the success of convolutional neural networks in the image domain, researchers started to apply CNNs to video tasks such as action recognition. However, ordinary convolutional neural networks cannot solve the video classification problem because both temporal and spatial features, spatiotemporal features, need to be extracted in video classification, while 2D convolutional neural networks can only extract spatial features of images, and for this reason, researchers have improved the traditional convolutional neural networks. There are three popular network models for video classification: (1) dual-stream network; (2) long and short-term memory network; (3) 3D convolutional neural network.

### 3.2. Combining 3D Convolutional for Action Recognition

3D convolutional neural network (3DCNN) was first proposed by Kai Yu et al. in 2013 for human behavior recognition, and then Du did an in-depth research and analysis on 3D convolutional neural network and proposed C3D network model and did a lot of experiments on the choice of convolutional kernel size, and the experiments proved that the convolutional kernel of size 3 × 3 × 3 achieved the best classification effect [22]. As the focus of vision tasks shifted from images to videos, researchers started to focus on 3D convolutional neural networks and applied the classical network structures of 2DC to 3DCNN, such as FVGG3D, Resnet3D, and Inception3D, in addition to FDensenet-3D, 13DF, and TemporalF3D. In 2015, NVIDIA Labs was the first to apply the C3D network model to action recognition, and the accuracy was significantly improved compared with the traditional vision-based action recognition algorithms. The main work of their paper has three points: (1) to prevent the overfitting of the network, they proposed some ways to augment the video data; (2) they designed two kinds of networks, high-resolution and low-resolution, and trained two subnetworks separately and finally fused them in the scoring layer; (3) they trained the network with RGB data and depth data and used two kinds of fusion, one is to train the network with RGB and depth separately, and then in 2017, NVIDIA labs fused RNN and 3DCNN into R3DCNN for action recognition, first extracting spatiotemporal features from short-time image sequences by 3DCNN and then regularizing these short-time spatiotemporal features by RNN to obtain long-time spatiotemporal features. This method is mainly applicable to very long image sequences or videos and finally achieves good results in their own datasets.

#### 3.2.1. 3D Convolutional Foundation Framework

The reason why ordinary convolutional neural networks can be successful in image tasks is that 2D convolutional kernels can extract spatial features of images very well. The 3D convolution kernel adds the temporal dimension to the 2D convolution kernel, and then 3D convolution is performed with the video block to extract the spatial and temporal features of the image sequence or video. The original image sequence or video is 3D convolved to generate feature cubes (2D convolution generates feature maps), and the feature cubes are then sequentially passed through subsequent 3D convolution layers to extract spatiotemporal features to generate new feature cubes.

The 3D convolutional neural network also requires downsampling, but the feature cube has replaced the feature map in the F2D convolution, so the 2D pooling layer is no longer applicable, so a new 3D pooling layer is introduced. 3D pooling increases the time dimension compared with 2D pooling and is used to downsample the length, width, and depth of the feature cube, which is still a feature cube after downsampling. The downsampling method used is still the same as the 2D pooling method. The most widely used is the maximum 3D pooling, which allows for displacement invariance in the selection of features from the extracted small feature cube and enhances the nonlinear fitting capability of the 3D convolutional network.

There is a very challenging problem in deep convolutional neural networks: gradient disappearance, which is generated by chaining the derivatives of the neural network during backpropagation and can slow down the convergence of the neural network leading to difficult training of the network. This problem has become a hot topic for researchers in the field of deep learning, and the ReLU function has alleviated this problem to some extent, and Kai-Ming He has introduced short connections in the proposed ResNet network structure, which makes the FF network still very efficient to train when it reaches 152 layers. However, the above two methods do not solve the problem from the perspective of training data [23]. The role of the Batch-Norm layer is to make the input data of each layer of the deep neural network obey the same distribution, more specifically; it transforms the input data to a normal distribution with mean *μ* and variance *σ*^2^. Due to the deep convolution network from shallow to deep and/or iterative optimization, the data distribution will shift to the saturated region at both ends of the nonlinear function (such as sigmoid function), and then do the back propagation chain derivation, and the generalized gradient will disappear. Therefore, after applying Batch-Norm, the input of each layer neuron will be forcibly changed from the saturated region after nonlinear mapping to the nonlinear unsaturated region, i.e., the region with larger gradient value, so as to avoid the problem of gradient disappearance.

#### 3.2.2. Multimodal Action Recognition

Currently, fusion of recognition results of multiple modalities to improve recognition rate has become the most common method in action recognition. The general method of multimodal fusion is to train the data of each modality separately to obtain recognition vectors and then fuse the recognition vectors of each modality by multiplying them together. In this way, there is no interaction between multiple modalities in the training phase, and the recognition results are only stacked, which is very limited in terms of accuracy improvement. In this paper, we propose a joint training approach for multiple modalities, which is divided into a training process and a recognition process.

Figure 7 shows the training process of our method. In the training phase, the RGB data are first fed into the 3D convolutional neural network built for training, and the specific parameters of the 3D convolutional neural network will be described later. After training, the convolutional neural network generates a network weight model, which stores the values of the convolutional kernels in each convolutional layer of the convolutional neural network. After training, the values of these convolutional kernels are saved as the weight model of the network. Note that the weight model at this point is only suitable for recognizing RGB data, but not for other modalities or the recognition rate is very low. However, we can fine-tune the RGB weight model with data from other modalities, which is a useful technique in convolutional neural networks. Simply put, fine-tuning is to apply the existing network structure of the network model to the dataset to be trained to achieve fast convergence. In many large-scale image recognition tasks, because the dataset is very large, it is often used a deep network structure such as VGG model, GoogLeNet, or ResNet, and if these networks are trained from scratch using the current dataset, not only is the convergence speed slow, but also the final recognition accuracy is very low. The network fine-tuning can be a good solution to this problem, because the features mentioned in the shallow layer of the deep convolutional neural network are some underlying visual features such as edges and textures, which are common features in many images, so the shallow convolutional kernel is usually frozen (no longer learning) when fine-tuning, and only the deep convolutional layer is trained, which will accelerate the convergence of the network.

Figure 8 illustrates the recognition process of our method. In the recognition phase, each modality is fed into the corresponding weight model to obtain the recognition vector of each modality (the probability of recognition into each class is stored in the vector), and then the recognition vectors of multiple modalities are multiplied to obtain the final recognition vector, and the index corresponding to the maximum value of the probability in the vector is the final classification result. At present, several strategies of fine-tuning are mainly based on the size relationship between the dataset of the entitled model and the dataset to be trained, as well as the similarity of the dataset. (1) The dataset to be trained is relatively small and the images are similar to the original dataset. (2) The dataset to be trained is large and the images are similar to the original dataset. (3) The dataset to be trained is small and the images are not similar to the original dataset. (4) The dataset to be trained is large but the images are not similar to the original dataset. Since we have a multimodal joint training, the number of samples in different modal datasets is the same and the contents are similar, so we can use the RGB weight model to fine-tune the whole network. When fine-tuning, a smaller learning rate should be used because the trained model weights and loss functions are already smoothed, and a larger learning rate will destroy the existing weights.

In our paper, instead of choosing the C3D network structure proposed by DuFTran, we designed a 3D convolutional neural network with 4 convolutional layers, 4 pooling layers, and 4 BN layers plus 2 fully connected layers, and the structure is shown in Figure 9. A single image is a plane, while a sequence of images or a video can be considered as a cube, and we can watch a video normally from the front of a cube to the back. But we can also choose to look from the left and top of the video, that is, from the left side of the cube to the right and above to the bottom. Although humans do not learn the content of the video by watching it in this way, due to the powerful learning ability of neural networks, they can learn different spatiotemporal features from different angles by learning from enough samples.

## 4. Experiments

### 4.1. Experimental Dataset and Network Parameters

We use our own collected dataset to evaluate our proposed method. The dataset contains a total of 1200 long jump samples, of which 900 samples are used for training and 300 samples are used for testing. Each sample contains both RGB and depth modalities and was acquired through a Microsoft Kinect device with an image resolution of 115 × 250. These samples were performed by eight peers and consisted of standing long jump and assisted long jump. The network parameters are shown in Table 1.

### 4.2. Key Frame Comparison Experiments

We have compared the key frame extraction based on uniform sampling and the key frame extraction based on optical flow on RGB data. After the statistics of video frames in the dataset, most of the video frames are in the range of 20–40 frames, so 16 frames, 24 frames, 32 frames, and 40 frames are selected, respectively, for the comparison experiments. When the total number of frames is less than 24, the video is expanded by using the random difference method, by first selecting a frame and then copying it and placing it behind the original image until it increases to 24; when the total number of frames is greater than 24 and less than 48, the frames in the video are randomly extracted and discarded until they are reduced to 24; when the number of frames is greater than 48, the video is sampled by setting a suitable interval to get 24 frames.

From Table 2, we can see that the accuracy rate increases to 53.2% with the increase of frame number from 16 to 24 to 32 frames but decreases instead of increasing after 40 frames. We guess that the main reason is that the total number of frames of some videos is less than 40, and these redundant frames affect the extraction of spatiotemporal features of long jump movements by the convolutional neural network after frame interpolation and augmentation, which leads to the decrease of accuracy.

We used the optical flow method to extract 16, 24, and 32 key frames from the video, and we did not conduct the experiment for 40 frames because we found that the recognition accuracy would be reduced when extracting 40 frames in the uniform sampling. Comparing Tables 2 and 3, we found that the accuracy of extracting 16, 24, and 32 key frames by optical flow method was significantly improved compared with the uniform sampling method, and the highest recognition rate was increased from 53.2% to 55.7%. Moreover, the accuracy rate is 52.6% when 24 frames are extracted by optical flow method, which indicates that the key frames extraction based on optical flow method can efficiently extract video frames with important motion information in the video.

### 4.3. Multimodal Training Experiments

We train and fine-tune the base of RGB, depth, and edge image models, respectively and compare the loss and accuracy difference between using fine-tuning and not using fine-tuning. Among them, the results of RGB image model are shown in Figure 10, the results of depth image model are shown in Figure 11, and the edge image model is shown in Figure 12. In the three experimental results, the red line is the network training directly using the original image, and the green curve is the fine-tuning on the basis of the original image model. It can be seen that if the training is done directly on the original image, it takes about 6000 iterations for the loss to approach convergence, while on the basis of fine-tuning training, it takes about 2500 iterations to converge. Therefore, using the fine-tuning method will greatly accelerate the convergence speed of the network.

Then, from Figure 10, the red curve is the accuracy curve of the directly trained deep image test set, and the green curve is the accuracy curve of the deep image test set based on the RGB training model; through comparison, it is found that, after using fine-tuning, not only is the convergence speed of the convergence network accelerated, but also the recognition accuracy is improved.

Then, we summarize the training accuracy results as Figures 13–15, where the red curve is the accuracy curve of the directly trained image model, and the green curve is the accuracy curve of the fine-tuning training based on the original image. By comparison, we found that, after using the fine-tuning, not only is the convergence speed of the convergence network accelerated, but also the recognition accuracy is improved to some extent.

Table 4 shows the recognition accuracy of different modalities and the comparison of the recognition accuracy of RGB, depth, and edge combination. From Table 4, it can be seen that the highest recognition accuracy of 75.4% was achieved for the edge images in the single modality comparison. Then, the recognition results of the three models were multiply fused and finally achieved 82.3% recognition accuracy, which is 6.9% higher than that of the edge images.

## 5. Conclusions

In this paper, from the perspective of rapid diagnostic feedback of students' physical health long jump test movements, we focus on realizing real-time and rapid processing and analysis capability of the video based on the reference of the previous kinematic analysis methods. In order to better analyze the long jump movements, we first use the video key frame extraction method of optical flow method and compare it with the video frame extraction based on uniform sampling method. The experiment proves that the optical flow method can indeed effectively extract the video frames with key movements in the video using motion information and improve the accuracy of recognition. Then, based on the 3D convolutional neural network, a multimodal joint training method for motion recognition is used. RGB images are trained on the 3D convolutional neural network to obtain the RGB weight model, while depth images and edge images are trained on the basis of the RGB weight model, and the recognition results of multiple modalities are fused. The system is stable, reliable, and easy to operate and can provide students with rapid diagnostic analysis of long jump technical movements and provide targeted advice for movement improvement. In the future, we plan to carry out research on long jump movement recognition based on graph convolution.

## Figures and Tables

**Figure 1:** Multimodal-based classification method for long jump technique.

**Figure 2:** Flowchart of vision-based action recognition.

**Figure 3:** Flowchart of contour-based action segmentation.

**Figure 4:** Tracking algorithm based on mean shift generative model.

**Figure 5:** Standard connection methods for fully connected layer.

**Figure 6:** Fully connected layer with dropout connection method.

**Figure 7:** Multimodal training flow.

**Figure 8:** Multimodal recognition process.

**Figure 9:** 3D convolutional neural network structure diagram.

**Figure 10:** Comparison of training loss before and after fine-tuning of RGB images.

**Figure 11:** Comparison of training loss before and after fine-tuning of depth images.

**Figure 12:** Comparison of training loss before and after fine-tuning of edge images.

**Figure 13:** Comparison of accuracy before and after fine-tuning of RGB images.

**Figure 14:** Comparison of accuracy before and after fine-tuning of depth images.

**Figure 15:** Comparison of accuracy before and after fine-tuning of edge images.

**Table 1:** Network parameter settings.

Parameters	Value
Learning rate	0.01
Momentum	0.9
Weight decay	0.0005
Minibatch	24
Gamma	0.9
Step size	[3000, 5000, 6500]
Maximum iteration	8850

**Table 2:** Accuracy of different frame rates under uniform sampling.

Number of frames	Accuracy (%)
16	46.5
24	49.7
32	53.2
40	51.4

**Table 3:** Accuracy of key frame extraction by optical flow method.

Number of frames	Accuracy (%)
16	48.9
24	52.6
32	55.7

**Table 4:** Accuracy of different modal types.

Modal type	Accuracy (%)
RGB	65.7
Depth	71.8
Edge	75.4
RGB + Depth + Edge	82.3

## Data Availability

The datasets used during the current study are available from the corresponding author on reasonable request.
